# Quercetin Alleviates Intervertebral Disc Degeneration by Modulating p38 MAPK-Mediated Autophagy

**DOI:** 10.1155/2021/6631562

**Published:** 2021-05-11

**Authors:** Shuwen Zhang, Weidong Liang, Yakefu Abulizi, Tao Xu, Rui Cao, Chuanhui Xun, Jian Zhang, Weibin Sheng

**Affiliations:** Department of Spine Surgery, The First Affiliated Hospital of Xinjiang Medical University, Urumqi 830054, China

## Abstract

Intervertebral disc degeneration (IVDD) is a degenerative and chronic spinal disorder often associated with the older population. Oxidative stress is a major pathogenic factor of aging that results in the apoptosis of nucleus pulposus cells (NPCs) and extracellular matrix (ECM) degradation. Quercetin (QUE), a naturally occurring flavonoid with antioxidant and anti-inflammatory properties, has been studied in research on degenerative diseases. However, the potential effects and mechanisms of action of QUE on IVDD remain unclear. In this study, the effects of QUE on antiapoptosis and ECM metabolism were firstly investigated in TBHP-treated NPCs. Meanwhile, the autophagy inhibitor, 3-MA, and p38 MAPK inhibitor, SB203580, were used in subsequent TBHP-induced NPC experiments to determine whether QUE exerted its protective effects through autophagy and the p38 MAPK/mTOR signaling pathway. Finally, the therapeutic effects of QUE were confirmed *in vivo* using a rat tail needle puncture-induced model of IVDD. We found that QUE treatment significantly alleviated oxidative stress-decreased cell viability and intracellular ROS levels in NPCs treated with TBHP. Furthermore, treatment with QUE led to a decrease in apoptosis as measured by decreased Bax and increased Bcl-2 expression and PE/7-AAD flow cytometry analysis. QUE also promoted ECM stability as measured by increased collagen II and aggrecan and decreased MMP13 levels. Our results also showed that QUE promoted the expression of autophagy markers beclin-1, LC3-II/I, and decreased p62. Inhibition of autophagy by inhibitor 3-MA may partially reverse the protective effect of QUE on apoptosis and ECM degeneration, indicating that autophagy was involved in the protective effect of QUE in NPCs. Further study confirmed that QUE partially inhibited the p38 MAPK signaling pathway and inhibition of p38 MAPK by SB203580 activated autophagy, indicating that QUE protected NPCs against apoptosis and prevented ECM degeneration via the p38 MAPK-autophagy pathway. Finally, using a rat tail puncture-induced model of IVDD, we confirmed that QUE had a protective effect against IVDD. Our results suggest that QUE could prevent IVDD by modulating p38 MAPK-mediated autophagy and, therefore, is a potential therapeutic strategy in the treatment of IVDD.

## 1. Introduction

Intervertebral disc degeneration (IVDD) is a degenerative disease that is the leading cause of lower back pain and disability and is therefore a significant health issue, especially in the elderly. Since approximately 80% of older people suffer from lower back pain, the aging population is contributing to an increased socio-economic burden on healthcare systems [1]. Due to the complexity of the spine, as well as the multiple factors that contribute towards IVDD pathogenesis, no effective conservative treatment is currently available. Most therapeutic strategies focus on symptomatic treatment or in the advanced stages of the disease, discectomy.

The physiological structure of nondegenerated intervertebral discs is maintained by the gelatinous nucleus pulposus (NP), external annulus fibrosus (AF), and the upper and lower cartilage endplates (CEP). It is well established that NP dysfunction is closely associated with IVDD. In NP tissue, nucleus pulposus cells (NPCs) play an important role in maintaining the homeostasis of the extracellular matrix (ECM). However, stimulation by external factors such as oxidative stress, inflammation, or mechanical loading, leads to increased apoptosis and catabolic/anabolic imbalances that eventually trigger and accelerate IVDD progression.

Excessive NPC apoptosis and ECM degradation caused by oxidative stress, inflammation, and mechanical loading are considered to be key pathogenic mechanisms of disc degeneration [2]. Oxidative stress has a pivotal role in the occurrence and progression of degenerative diseases, and the overproduction and/or reduced clearance of reactive oxygen species (ROS) may be a potential therapeutic target for IVDD [3]. Both oxidative stress and its ROS by-products increase with aging and are closely associated with the degree of disc degeneration by promoting apoptosis and impeding ECM metabolism [4–6]. Tert-butyl hydroperoxide (TBHP) is an exogenous inducer of oxidative stress and has been previously used in models of degenerative diseases such as osteoarthritis due to its high stability and sustained release capability [7]. Here, we used TBHP to establish a stable oxidative stress model in NPCs.

Quercetin (QUE), a member of the natural flavonoid family, has antioxidative stress, antiapoptosis, and anti-inflammatory properties [8, 9]. Recent studies have shown that QUE could have therapeutic effects on the liver, kidneys, cardiovascular system, and in degenerative disorders by modulating the SIRT1, AMPK, and MAPK signaling pathways [10–12]. QUE has recently been used to treat osteoarthritis based on its ability to inhibit apoptosis, which modulates AMPK-mediated endoplasmic reticulum stress [13]. However, it remains unclear whether these pathways have a role in the regulation of autophagy. Furthermore, little is known about the potential therapeutic role of QUE in the regulation of autophagy, especially in IVDD.

Autophagy is a conserved cellular degradation process that mediates intracellular homeostasis and protects cells against stresses by degrading and recycling dysfunctional or damaged proteins and organelles [14]. Although preliminary studies have examined the causal relationship between autophagy and IVDD, further work is required to understand its complex mechanism and potential therapeutic targets [15]. The MAPK pathway is an upstream regulator of autophagy [16, 17]. Specifically, the p38 MAPK signaling pathway, which modulates cellular processes, such as proliferation, differentiation, and survival and death, has been associated with oxidative stress and aging-related diseases [18]. The p38 MAPK signaling pathway, activated by cellular stress such as cell damage, regulates intracellular homeostasis [19]. *In vivo* and *in vitro* experiments have confirmed that phosphorylation of p38 MAPK induces apoptosis and increases tissue inflammation [19, 20].

Based on these studies, we hypothesized that QUE could attenuate IVDD through the suppression of NPC apoptosis and ECM degradation by regulating autophagy in a p38 MAPK-dependent manner. TBHP-treated NPCs and an in vivo needle-punctured rat tail model were used as models of IVDD to examine the protective effect of QUE on IVDD.

## 2. Material and Methods

### 2.1. NPC Isolation and Culture and Experimental Design

Primary NPCs were isolated from the NP tissue of 4-week-old Sprague-Dawley (SD) rats (specific pathogen-free). The NP tissue pieces were digested in 0.2% type II collagenase (Solarbio, Beijing, China) for 25 min at 37°C, filtered through a 0.75 *μ*m cellular filter, resuspended in DMEM/F12 with 12% fetal bovine serum (Hyclone, USA) and 1% antibiotics, then placed in a 5% CO_2_ incubator at 37°C. NPCs were subcultured when they reached 80%–90% confluence. The first three passages of NPCs were used for all experiments.

Oxidative stress was induced in NPCs by treatment with TBHP (50 *μ*M) for 24 h. In experiments that examined the effects of QUE, NPCs were pretreated with QUE (15 *μ*M or 25 *μ*M) for 2 h before induction of oxidative stress with TBHP (50 *μ*M). The autophagy inhibitor 3-MA was purchased from Selleck USA and used at a concentration of 10 mM. The p38 MAPK inhibitor was obtained from Selleck USA and used at a concentration of 10 *μ*M.

### 2.2. Cell Viability Assay

Cell viability was measured using the cell counting kit-8 (Bioss, Beijing, China) according to the manufacturer's instructions. NPCs were seeded in 96-well plates at a density of 5 × 10^3^ cells/well and incubated with different concentrations of QUE and TBHP for 24 h. CCK8 solution (10 *μ*l) was added to each well, and NPCs were cultured for a further 1–2 h at 37°C. The absorbance of each sample was measured at 450 nm using a microplate reader (Thermo, USA).

### 2.3. Flow Cytometric Analysis of ROS

Intracellular ROS was detected using a ROS assay kit (Solarbio). Briefly, the treated NPCs were incubated with 10 *μ*M fluorescent 2,7-dichlorodihydro-fluorescein diacetate (DCFH-DA) at 37°C and mixed by inversion every 3–5 min for 30 min. NPCs were then washed three times with cold DMEM/F12 and analyzed by flow cytometry (BD Biosciences, USA).

### 2.4. Flow Cytometric Analysis of Apoptosis

NPCs were labeled by double staining with an annexin V-phycoerythrin (PE)/7-aminoactinomycin (7-AAD) Kit (BD Biosciences, USA). Treated NPCs were collected, washed three times with cold phosphate-buffered saline (PBS), resuspended in 100 *μ*l 1× binding buffer (1 × 10^5^ cells), and incubated with 5 *μ*l Annexin V-PE and 5 *μ*l 7-AAD for 15 min at room temperature in the dark. The stained NPCs were diluted with 400 *μ*l 1× binding buffer and counted by flow cytometry (BD Biosciences, USA).

### 2.5. Immunofluorescence Staining

NPCs were cultured in 35 mm glass culture dishes and treated with different interventions for 24 h according to the experimental design. NPCs were then washed with cold PBS, fixed in 4% paraformaldehyde for 15–30 min, permeabilized with 0.5% Triton X-100 for 20 min, and blocked with 5% bovine serum albumin (BSA) for 1 h at 37°C. Next, samples were incubated with primary antibodies against collagen II (1 : 100; Abcam, UK) and MMP13 (1 : 50; Abcam, UK) overnight at 4°C. The following day, samples were incubated with Alexa Fluor®488 or 594-labeled goat anti-rabbit IgG antibody (1 : 100) for 1 h at room temperature, then labeled with diamidino-2-phenylindole for 5–10 min. Finally, samples were observed under a confocal fluorescence microscope (Leica, Germany), and the fluorescence intensity was analyzed by Image J software 2.1 (Bethesda, MD, USA).

### 2.6. Western Blot Analysis

NPCs were lysed using RIPA buffer (Thermo, USA) containing protease and phosphatase inhibitors (with a ratio volume of 100 : 1). Samples were quantified using a BCA protein assay kit (Thermo, USA). Equal amounts of total protein for each treatment group were separated by SDS-PAGE gel and transferred to a polyvinylidene difluoride membrane. After blocking with 5% nonfat milk or 5% BSA for 2 h at room temperature, the membranes were incubated overnight at 4°C with primary antibodies against Bcl 2 (1 : 1000, Proteintech, China), BAX (1 : 2000, Proteintech), collagen II (1 : 1000, Abcam, UK), MMP13 (1 : 2500, Bioss, China), aggrecan (ACAN, 1 : 1000, Proteintech), p38MAPK (1 : 1000, CST, USA), p-p38MAPK (1 : 1000, CST), p-mTOR (1 : 1000, CST), mTOR (1 : 1000, CST), LC3 II/I (1 : 1000, CST), Beclin-1 (1 : 1000, CST), p62 (1 : 1000, CST), and GAPDH (1 : 5000, Proteintech). The next day, membranes were incubated with HRP-conjugated secondary antibodies (1 : 5000, ZSGB-BIO, China) for 2 h at room temperature. Protein bands were detected with enhanced chemiluminescence (Biosharp, China) and quantified using Image Lab software (Bio-Rad, USA).

### 2.7. Transmission Electron Microscopy (TEM)

To observe the autophagosomes and autophagolysosomes, treated NPCs were fixed overnight in 2.5% glutaraldehyde, postfixed in 2% osmium tetroxide for 1 h, and resuspended in fetal bovine serum. After washing, samples were dehydrated with graded acetone solutions, embedded in epoxy resin, cut into ultrathin sections, and stained with saturated uranyl acetate-lead citrate. Sections were visualized using a transmission electron microscope (Hitachi, Japan).

### 2.8. Surgical Procedure and Rat IVDD Model

A total of 36 male SD rats, aged 8 weeks, weighing between 200 and 250 g, were randomly assigned to the following groups: group I was the control group (control, *n* = 12), group II was the puncture and saline treatment group (saline, *n* = 12), and group III was the puncture and QUE treatment group (QUE, *n* = 12).

To induce IVDD, rats were anesthetized intraperitoneally with pentobarbital (40 mg/kg), after which their tail skin was sterilized with iodine solution and punctured to the AF layer with 27-gauge sterile needles. The puncturing process was confirmed using a portable high-frequency X-ray unit (Erlang Sense, China). All needles were kept in position about 4 mm from the skin for 1 min after the needle had rotated 360° [21]. After surgery, QUE (100 mg/kg) was administered intragastrically once a day to the group III rats while the group II rats received the same volume of saline daily for the time course of the experiment. All experimental protocols were performed according to the Declaration of Helsinki and the Guide for Care and Use of Laboratory Animals and were approved by the Animal Ethics Committee of Xinjiang Medical University Animal Center (IACUC-20190225-22).

### 2.9. Magnetic Resonance Imaging (MRI)

At 0, 4, and 8 weeks after the puncture-induced IVDD procedure, rats were anesthetized and examined using a 3.0 MRI system (MRI, Siemens, Germany). Sagittal T2-weighted parameters were set as follows: fast-spin echo sequence with time to repetition of 5400 ms and time to echo of 236 ms, 320 (h) 9 256 (v) matrix, field of view of 200, 4 excitations, and slice thickness of 1.6 mm. The degree of IVDD was assessed in accordance with the Pfirrmann grading of T2-weighted images (1, 2, 3, and 4 points indicated grades I, II, III, and IV, respectively).

### 2.10. Histological Analysis

Eight weeks after the puncture procedure, rat tails were collected and fixed in 4% formaldehyde for 48 h, then decalcified for 1 month. Tails were then dehydrated in gradient alcohol, embedded in Leica paraffin, and cut into 4 *μ*m sections. The serial sections of each sample were stained with Hematoxylin and Eosin (H&E), Safranin-O/Fast Green, and Alcian blue. An improved histopathological grading score system was used to evaluate the degree of degeneration of the intervertebral discs in each group according to the cellularity and morphology of the NPCs and AFCs and the border between the NP and AF (5, 6–11, and 12–14 scores indicate normal discs, moderately degenerated discs, and severely degenerated discs, respectively).

### 2.11. Immunohistochemical Staining

ACAN, Bax, and Beclin1 expression levels were detected using immunohistochemical staining. Briefly, paraffin slices of intervertebral disc tissue were heated for 2 h at 60°C, dewaxed in xylene for 30 min, dehydrated in graded ethanol for 5 s, and blocked with 3% H_2_O_2_ for 10 min. Slices were then washed in PBS for 15 min, incubated with 0.4% pepsin in 5 mM HCL for antigen retrieval for 30 min at 37°C, and blocked with goat serum for 30 min at room temperature. Next, the slices were incubated with primary antibodies against ACAN (1 : 200, Proteintech, China), Bax, (1 : 400, Proteintech), and Beclin1 (1 : 200, CST, USA) overnight at 4°C. The next day, the slices were washed three times with PBS for 15 min and incubated with HRP-conjugated secondary antibody for 2 h at room temperature. The slices were stained with 3, 3-diaminobenzidine, counterstained with hematoxylin, dehydrated with graded ethanol, and analyzed by light microscopy (Leica, Germany).

### 2.12. Statistical Analysis

Experimental data from 3 replicates are presented as the mean ± standard deviation. SPSS 26.0 (SPSS Inc, Chicago, USA) was used to perform one-way analysis of variance (ANOVA) followed by Tukey's test to determine statistical significance among different groups. Pfirrmann grading and histological score were analyzed by the Kruskal-Wallis H test. *P* value < 0.05 indicated statistical significance between groups.

## 3. Results

### 3.1. The Effects of QUE and TBHP on the Viability of NPCs

As shown in Figure 1(a), the growth curve indicates that NPCs were in the logarithmic phase during the first 24 h of culture. The cytotoxicity of QUE and TBHP on NPCs was determined at gradient concentrations (QUE: 0, 15, 25, 50, 75, 100, and 200 *μ*M) and (TBHP: 0, 5, 15, 25, 50, 100, and 200 *μ*M) for 24 h. We found that cell viability was reduced at concentrations of QUE greater than 50 *μ*M, whereas lower concentrations of QUE (15 *μ*M and 25 *μ*M) had no cytotoxic effects on NPCs after 24 h (Figure 1(b)). Cell viability was markedly decreased after treatment with 50 *μ*M TBHP for 24 h (Figure 1(c)), while pretreatment with 25 *μ*M QUE reversed this TBPH-induced cytotoxic effect (Figure 1(d)). Changes in cell morphology including cell shrinkage and vacuole formation were observed in 50 *μ*M TBHP-treated NPCs, whereas pretreatment with QUE was found to alleviate the morphological changes induced by TBHP (Figure 1(e)).

### 3.2. QUE Protects NPCs against TBHP-Induced Apoptosis and ECM Degradation

Flow cytometric analysis of DCF intensity was used as a measure of intracellular ROS levels. We found that intracellular ROS levels were significantly increased when NPCs were treated with TBHP. However, pretreatment with QUE significantly reduced TBHP-induced ROS production in NPCs (Figures 2(a) and 2(b)). Western blot analysis was performed to evaluate the protective effect of QUE on TBHP-treated NPCs. NPCs were pretreated with 15 *μ*M or 25 *μ*M QUE for 2 h before TBHP simulation for 24 h. We found that TBHP treatment significantly decreased Bcl-2 levels, while increasing Bax expression. These effects were reversed by pretreatment with QUE (Figures 2(c) and 2(d)). As shown in Figures 2(c) and 2(d), the ECM was disrupted after treatment with 50 *μ*M TBHP, as measured by decreased collagen II and ACAN protein expression, and increased MMP13 levels. Pretreatment with QUE increased collagen II and ACAN expression and suppressed MMP13 expression.

### 3.3. QUE Treatment Upregulates Autophagy in NPCs

To determine the effect of QUE on autophagy, NPCs were pretreated with 3-MA, an autophagy inhibitor, before administration of QUE and TBHP. As shown in Figures 3(a) and 3(b), QUE treatment resulted in upregulation of Beclin-1 and the LC3 II/I ratio and a decrease in p62 protein expression in TBHP-treated NPCs. Compared with the QUE group, pretreatment with 10 mM 3-MA led to a decrease in Beclin-1 and LC3 II/I but had little effect on p62 expression. TEM revealed that QUE pretreatment of TBHP-treated NPCs led to an increase in autophagosomes and autophagolysosomes, whereas a decreased number of autophagosomes were observed after treatment with 3-MA (Figure 3(c)). Thus, our findings suggest that QUE upregulates autophagy in our TBHP-induced NPC model of IVDD.

### 3.4. QUE Protects against Apoptosis and ECM Degradation via Upregulation of Autophagy in TBHP-Treated NPCs

To further understand the relationship between autophagy and the antiapoptotic effects of QUE, NPCs were pretreated with 3-MA before treatment with QUE in TBPH-treated NPCs. We found that 3-MA pretreatment blocked autophagy (Figure 3), decreased Bcl-2 protein levels, and increased Bax expression (Figures 4(a) and 4(b)). Consistent with these findings, flow cytometry analysis revealed that TBHP-induced NPC apoptosis was markedly decreased in the presence of QUE, but this effect was reversed by pretreatment with 3-MA (Figures 4(c) and 4(d)). As shown in Figures 5(a) and 5(b), TBHP significantly downregulated the protein expression of collagen II and ACAN, while it upregulated MMP13 levels, suggesting that QUE could protect against ECM degradation. However, pretreatment with 3-MA reversed this protective effect of QUE. Consistent with these findings, immunofluorescence staining indicated that the role of QUE in maintaining the ECM metabolic balance was weakened by the autophagy inhibitor 3-MA (Figures 5(c)–5(f)).

### 3.5. QUE Activates Autophagy by Modulating the p38MAPK/mTOR Signaling Pathway in TBHP-Treated NPCs

To determine whether QUE is involved in regulating the p38MAPK signaling pathway in TBHP-treated NPCs, changes in p38MAPK activation were examined by analyzing the phosphorylation status of p38MAPK by Western blot. The increase in p38MAPK phosphorylation that was observed in NPCs after treatment with TBHP was reduced by QUE pretreatment (Figures 6(a) and 6(b)). Next, SB203580, a p38MAPK inhibitor, was used to examine the effect of QUE on the p38MAPK/mTOR signaling pathway. As expected, both QUE and SB203580 inhibited the phosphorylation of p38MAPK and mTOR (Figures 6(a) and 6(b)). Finally, SB203580 was used to test the hypothesis that QUE mediated autophagy via the p38MAPK/mTOR signaling pathway. As shown in Figures 6(c) and 6(d), both QUE and SB203580 (10 *μ*M) could activate autophagy. Taken together, our findings demonstrated that QUE ameliorates autophagy by inhibiting TBHP-induced p38MAPK/mTOR activation in rat NPCs, resulting in decreased cell apoptosis and ECM degradation.

### 3.6. QUE Attenuates IVDD in the Puncture-Induced Rat Tail Model of IVDD

The effects of QUE in IVDD was next investigated using the rat tail puncture model. The Pfirrmann grade, which measures the severity of disc degeneration (according to MRI T2-weighted signal intensity), was lower in QUE-treated puncture-induced rats than saline-treated controls 4 and 8 weeks postsurgery (Figures 7(a) and 7(b)). H&E staining revealed that the histological structure of the NP had almost disappeared and that the AF had bulged inwards and ruptured, while the border between the NP and AF was severely disrupted in the saline-treated control group 8 weeks after induction of IVDD. However, QUE treatment alleviated the degeneration and morphological changes in NP and AF (Figures 7(c) and 7(d)). Both Safranin-O/Fast Green and Alcian blue staining indicated that ECM proteoglycans were better preserved in the QUE group compared with the saline group 8 weeks after puncture (Figure 7(c)). Finally, immunohistochemical staining revealed that QUE treatment increased ACAN (Figure 8(a)) and Beclin1 (Figure 8(c)) expression and decreased Bax levels (Figure 8(b)) in the degenerative rat discs. Taken together, our findings indicate that QUE exerts an antiapoptotic effect in our *in vivo* model of IVDD.

## 4. Discussion

Currently, pharmacological treatment strategies for degenerative disc disease aim to alleviate the patients' symptoms. However, they fail to control or reverse the progression of IVDD and cause some side effects [1, 22]. Surgery is required at an advanced stage of IVDD when conservative treatment fails, and this is accompanied by various surgical risks [23]. Thus, the development of an effective drug that would prevent or alleviate the progression of IVDD is crucial. In recent years, natural herbal extracts have been used to treat clinical illnesses due to their antiapoptotic and anti-inflammatory effects and minimal side effects [7, 24–27]. Here, we show that treatment with QUE, a naturally occurring flavonoid, inhibits apoptosis and attenuates ECM degradation via autophagy in TBHP-induced NPCs. In addition, our *in vivo* study confirms the protective effect of QUE in a tail puncture-induced IVDD rat model.

Excessive apoptosis in intervertebral disc cells, especially NPCs, leads to changes in intervertebral disc structure and function and is one of the most important pathophysiological mechanisms underlying IVDD progression [2]. Apoptosis is a complex phenomenon involving multiple inducing factors, such as oxidative stress and inflammation. Oxidative stress, also thought to be associated with cell apoptosis, is closely associated with the occurrence and development of aging and degenerative diseases [3]. Physiologically, ROS is formed as a normal by-product of oxygen metabolism and has a pivotal role in homeostasis and cell signaling [28]. However, excessive ROS has been reported in the pathogenesis of IVDD, resulting in induction of NPC apoptosis and ECM degradation [4, 29]. Studies have confirmed that both TBHP and H_2_O_2_ could induce apoptosis of NPCs and metabolic imbalance of the ECM by producing large amounts of ROS [7, 30].

Previous studies have suggested that the ECM is maintained by both synthesis and catabolism and that disruption of either process affects the structure and functionality of the ECM [31]. The synthesis and degradation of the ECM in healthy intervertebral discs maintain a dynamic balance, especially in NPCs. Oxidative stress, however, disrupts this homeostasis by increasing secretion and expression of proteases such as MMPs and ADAMTs and downregulating expression of ECM proteins such as collagen II and ACAN [32]. Thus, oxidative stress-induced DNA damage in NPCs reduces their ability to synthesize ECM components, while increasing the production of matrix metalloproteinases, which promote catabolism of the ECM. Our results were consistent with these previous studies.

Autophagy is essentially a lysosome-mediated intracellular catabolic process in which dysfunctional cytoplasmic macromolecules and damaged organelles can be degraded and recycled in response to external stimuli to increased metabolism. Previous studies have confirmed the relationship between autophagy and IVDD [33]. Low levels of autophagy are found in healthy intervertebral discs. Autophagy is activated in mild IVDD, but decreased in severe IVDD. Previous studies have demonstrated that activation of autophagy could protect cells against apoptosis [34]. Specifically, natural small molecule compounds that regulate autophagy were reported to inhibit the oxidative stress-induced apoptosis of NPCs and degradation of the ECM and to reduce the progression of IVDD induced by tail puncture [7, 26, 30].

QUE, a ubiquitous flavonol derived from rutin, hawthorn, bupleurum, and onion, has been reported to inhibit oxidative stress and inflammation in degenerative diseases with minor side effects [8, 35, 36]. Previous studies have verified the therapeutic effects of QUE on different regulatory mechanisms in other diseases [13, 36, 37]. Recent studies have confirmed that QUE could alleviate osteoarthritis through regulating dysfunctional mitochondria or endoplasmic reticulum, which are involved in attenuating ROS levels and inhibiting chondrocyte apoptosis through upregulation of SIRT1 and phosphorylation of AMPK [13, 38]. Studies have also confirmed that the antiapoptotic effect of QUE is associated with the MAPK signaling pathway. One study revealed that pretreatment with QUE significantly reduced the expression of Bax, caspase-3, and cytochrome c and increased expression of Bcl-2 in lipopolysaccharide-induced MC3T3-E1 cells [39]. Both the AMPK and MAPK signaling pathways are closely associated with autophagy. Here, TEM revealed that QUE activated autophagy in TBHP-treated NPCs. p62 expression was significantly increased in TBHP-treated NPCs, indicating that the degradation of autophagosomes was inhibited, that is, the autophagy flux process was blocked. However, pretreatment with QUE appeared to reverse this phenomenon. Furthermore, pretreatment with the autophagy inhibitor, 3-MA, inhibited autophagy formation, but had virtually no blocking effect on the degradation of autophagolysosomes, as measured by little increased protein levels of p62 and a decreased ratio of LC3-II/I. In this study, QUE combined with 3-MA reduced the protective effect of QUE treatment alone on TBHP-induced oxidative stress in NPCs, suggesting that QUE activates autophagy to prevent apoptosis and ECM degradation.

p38 MAPK, a major signal transduction pathway, is closely correlated with the pathogenesis of IVDD [40]. p38 MAPK can be activated by environmental stimuli, such as inflammatory factors and oxidative stress, and regulates mTOR directly [29, 41]. p38 MAPK phosphorylation was increased in degenerative disc tissue compared with normal tissue and may be involved in the regulation of cellular processes such as cell proliferation, differentiation, inflammation, and apoptosis [18, 42]. Little is known about whether the protective effect of QUE on IVDD is mediated via the p38 MAPK signaling pathway. Here, we found that both p38 MAPK and mTOR were activated in TBHP-treated NPCs. Pretreatment with QUE or the p38 MAPK inhibitor SB203580 decreased the phosphorylation of p38 MAPK and partially decreased phosphorylation of mTOR. Thus, our data suggest that QUE acts via the p38 MAPK/mTOR signaling pathway.

We next sought to determine whether the protective effect of QUE on IVDD was mediated through p38MAPK-dependent autophagy using the p38 MAPK inhibitor, SB203580, and measuring autophagy-related protein expression levels. As expected, both QUE and SB203580 treatment led to an increase in Beclin1 and LC3II/I expression while p62 levels were decreased. Interestingly, slightly higher levels of autophagy were observed after QUE treatment than SB203580. This may be because QUE could directly or indirectly regulate autophagy through other signaling pathways. Aysa et al. [36] reported that QUE alleviates high glucose-induced damage on umbilical vein endothelial cells by promoting autophagy, although the specific autophagy-related pathways were not analyzed. Recently, QUE has been shown to suppress apoptosis and attenuate IVDD via the SIRT1-autophagy pathway [43], while He et al. [9] reported that QUE could induce autophagy via the FOXO1-dependent pathways. Taken together, these studies suggest that in addition to the p38 MAPK pathway, QUE may, at least partially, reduce the oxidative stress-induced injury of NPCs through these additional pathways. In addition, both MR imaging and histological results indicated that QUE could ameliorate the progression of IVDD *in vivo.* Moreover, QUE treatment suppressed the apoptotic protein Bax and promoted autophagy maker Beclin1 in degenerative discs.

## 5. Conclusion

In summary, our current study suggests that QUE protects against TBHP-induced NPC apoptosis and ECM degradation via autophagy activation mediated by suppressing the p38 MAPK/mTOR signaling pathway. Furthermore, QUE attenuated IVDD in a rat tail puncture-induced model, showing the potential value of QUE for the treatment of IVDD.

## Figures and Tables

**Figure 1:** The effects of QUE and TBHP on NPC viability. (a) Growth curves of NPCs during the first 72 h of culture. (b, c) Viability of NPCs treated with different concentrations of QUE and TBHP for 24 h. (d) Viability of TBHP-induced NPCs pretreated with QUE. (e) Representative images showing morphological changes in NPCs after pretreatment with different concentrations of QUE followed by incubation with 50 *μ*M TBHP (original magnification ×200, scale bar: 50 *μ*m). Data are presented as mean ± standard deviation from three independent experiments. ^#^*P* < 0.01 vs. control group; ^∗^*P* < 0.05 and ^∗∗^*P* < 0.01 vs. TBHP-induced group.

**Figure 2:** QUE protects NPCs against TBHP-induced apoptosis and ECM degradation. (a) Measurement of intracellular ROS levels by flow cytometry. (b) Quantification of ROS levels by measuring the DCFH-DA fluorescence intensity in each treatment group. (c) Western blot analysis of the prosurvival protein, Bcl-2, and proapoptotic protein, Bax, and ECM-related proteins, collagen II, ACAN, and MMP13. (d) Quantification of protein levels for Bcl 2, Bax, collagen II, ACAN, and MMP13. Data are presented as the mean ± standard deviation from three independent experiments. ^∗^*P* < 0.05; ^∗∗^*P* < 0.01; ^∗∗∗^*P* < 0.001.

**Figure 3:** QUE treatment upregulates autophagy in NPCs. (a) Western blot analysis of the autophagy-related proteins, Beclin-1 and p62, and LC3 II/I. (b) Quantification of Beclin-1, p62, and LC3 II/I protein levels. (c) Representative TEM image showing the autophagic changes in NPCs after various treatments. Black arrow: autophagosome; white arrow: autophagolysosome. Original magnification ×30000, scale bar: 500 nm. Data are presented as mean ± standard deviation from three independent experiments. ^∗^*P* < 0.05; ^∗∗^*P* < 0.01; ^∗∗∗^*P* < 0.001.

**Figure 4:** Pretreatment with 3-MA reverses the antiapoptotic effects of QUE on TBHP-treated NPCs. (a) Western blot analysis of the prosurvival (Bcl-2) and proapoptotic (Bax) proteins. (b) Quantification of the protein levels of Bcl-2 and Bax. (c) Apoptotic NPCs were stained with Annexin V PE/7-AAD double-fluorescence and analyzed by flow cytometry. (d) Quantification of the apoptotic rate based on the flow cytometry data. Data are presented as mean ± standard deviation from three independent experiments. ^∗^*P* < 0.05; ^∗∗^*P* < 0.01; ^∗∗∗^*P* < 0.001.

**Figure 5:** QUE regulates the ECM metabolic balance via autophagy in TBHP-treated NPCs. (a) Western blot analysis of the ECM components, collagen II and ACAN, and the degrading enzyme, MMP13. (b) Quantification of collagen II, ACAN, and MMP13 protein levels. (c, d) Representative images showing immunofluorescence staining for collagen II and MMP13 (collagen II: Alexa Fluor®488 labeled secondary antibody; MMP13: Alexa Fluor®594 labeled secondary antibody, original magnification ×200, scale bar: 75 *μ*m). (e, f) Semiquantitative analysis of collagen II and MMP13 immunofluorescence staining. Data are presented as mean ± standard deviation from three independent experiments. ^∗^*P* < 0.05; ^∗∗^*P* < 0.01; ^∗∗∗^*P* < 0.001.

**Figure 6:** QUE activates autophagy via inhibition of the p38MAPK/mTOR signaling pathway. (a) Western blot analysis of the p38 MAPK/mTOR signaling pathway components, p-p38, p38, p-mTOR, and mTOR in TBHP-induced NPCs treated with QUE or the p38 MAPK inhibitor, SB203580. (b) Quantification of p-p38 and p-mTOR protein levels. (c) Western blot analysis of the autophagy-related proteins, Beclin-1, p62, and LC3 II/I in TBHP-induced NPCs treated with QUE or SB203580. (d) Quantification of Beclin-1, p62, and LC3 II/I protein levels. Data are presented as mean ± standard deviation from three independent experiments. ^∗^*P* < 0.05; ^∗∗^*P* < 0.01; ^∗∗∗^*P* < 0.001.

**Figure 7:** QUE attenuates the progression of IVDD in the rat tail needle puncture-induced IVDD model. (a) Representative T2-weighted images of MRI scans for the needle-punctured discs 4 and 8 weeks postsurgery (red boxes indicate the punctured level). (b) Pfirrmann grade scores based on the MRI T2-weighted signal intensity 4 and 8 weeks postsurgery. (c) Representative H&E images showing the histopathology and cell morphology and Safranin-O/Fast Green and Alcian blue staining showing proteoglycan deposition in different experimental groups 8 weeks postsurgery (original magnification ×25, scale bar: 500 *μ*m). (d) The improved histopathological grading score of intervertebral discs were calculated for each group. Data are presented as mean ± standard deviation from three independent experiments. ^#^*P* < 0.01 vs. control group, ^∗^*P* < 0.05; ^∗∗^*P* < 0.01 vs. saline group.

**Figure 8:** Mechanisms of QUE on the treatment of IVDD. (a) Immunohistochemical staining of the ECM-related protein ACAN in the disc sections 8 weeks postsurgery (original magnification ×25 or ×200). (b) Immunohistochemical staining of the proapoptotic protein Bax in the disc sections 8 weeks postsurgery (original magnification ×25 or ×200). (c) Immunohistochemical staining of the autophagy-related protein Beclin1 in the disc sections 8 weeks postsurgery (original magnification ×25 or ×200).

## Data Availability

The data that support the findings of this study are available on request from the corresponding author.
